The article "Anaesthesia in on-pump cardiac surgery for congenital heart diseases at the Cuomo Pediatric Cardiology Center (Senegal)" was retracted in 2021. Reason: duplicate publication.

# Prise en charge anesthésique des cardiopathies congénitales opérées sous circulation extra - corporelle au Centre de Chirurgie Cardiaque Pédiatrique Cuomo (Sénégal)

**DOI:** 10.11604/pamj.2020.37.362.17659

**Published:** 2020-12-21

**Authors:** Farid Pingwindé Belem, El Hadji Boubacar Ba, Papa Alassane Leye, El Hadji Ndiassé Diop, Ibrahima Gaye, Mamadou Diawo Bah, Etienne Birame Sène, Marie Victoire Sène, Mohamed Lamine Fall, Amadou Gabriel Ciss, Oumar Kane

**Affiliations:** 1 Service d´Anesthésie - Réanimation, CHU de Fann, Dakar, Sénégal,; 2 Service d´Anesthésie - Réanimation, CHU Aristide Ledantec, Dakar, Sénégal,; 3 Service de Chirurgie Thoracique et Cardiovasculaire, CHU de Fann, Dakar, Sénégal

**Keywords:** Cardiopathies congénitales, anesthésie, circulation extra-corporelle, Congenital heart diseases, anesthesia, on-pump cardiac surgery

## Abstract

Les cardiopathies congénitales surviennent dans 0,5 - 1% des naissances. La prise en charge d´enfants souffrant de malformation cardiaque nécessite un centre adapté, un matériel médical adéquat et des connaissances particulières tant sur le plan anesthésique que chirurgical. L´objectif de ce travail était d´évaluer la prise en charge anesthésique de ces cardiopathies dans notre centre après une première année d´activité et de comparer les résultats obtenus aux données de la littérature. Nous avons mené une étude rétrospective, descriptive sur une année allant de janvier à décembre 2017. Ont été inclus tous les patients opérés au cours de cette période pour une cure de cardiopathie congénitale sous circulation extracorporelle. Nous avons colligé 80 dossiers de patients opérés pour une cardiopathie congénitale. Parmi ces 80 patients, 60 ont été opéré sous circulation extra corporelle (CEC) soit un taux de 75%. L´âge moyen de nos patients était de 7,41 ans avec un sex- ratio de 1,22. La durée de la CEC était en moyenne de 82,82 mn et la durée moyenne du clampage aortique était de 58,31 mn. Soixante-dix pourcent (70%) des patients ont eu des catécholamines en fin d´intervention. La complication la plus fréquente en post opératoire était la défaillance cardiaque droite (69%). La durée moyenne de séjour en réanimation était de 4,33 jours. Nous avons noté le décès d´un patient portant la mortalité à 1,6%. Les cardiopathies congénitales sont complexes et très variables. Avec l´amélioration des techniques de prise en charge, leur morbi-mortalité a fortement diminué.

## Abstract (en)

Congenital heart diseases account for 0.5-1% of births. The management of children with cardiac malformation requires treatment in a suitable center, adequate medical equipment and specific anesthetic and surgical knowledge. The purpose of this study was to evaluate the anesthetic management of patients with congenital heart diseases in our center after the first year of activity and to compare the obtained results with literature reported data. We conducted a retrospective, descriptive study over a 1-year period, from January to December 2017. All patients undergoing on-pump cardiac surgery for congenital heart disease during this period were included. We collected data from 80 records of patients undergoing surgery for congenital heart disease. Out of these 80 patients, 60 underwent on-pump cardiac surgery (75%). The average age of patients was 7.41 years, with a sex-ratio of 1.22. The mean duration of on-pump cardiac surgery was 82.82 min and the mean duration of aortic clamping was 58.31 min. At the end of the procedure catecholamine production was found in 70% of patients. The most common complication in the postoperative period was right-side heart failure (69%). The average length of stay in the Emergency room was 4.33 days. One patient died, bringing mortality to 1.6%. Congenital heart diseases are complex and highly variable. Improved management techniques have strongly reduced morbi-mortality.

The article "Anaesthesia in on-pump cardiac surgery for congenital heart diseases at the Cuomo Pediatric Cardiology Center (Senegal)" was retracted in 2021. Reason: duplicate publication.

## Introduction

Les cardiopathies congénitales sont assez fréquentes. Elles surviennent dans 0,5 - 1% des naissances [1]. Bien que d´innombrables malformations aient été décrites, les trois quarts d´entre elles font partie des anomalies suivantes: communication inter - ventriculaire (CIV), persistance du canal artériel (PCA), communication inter- auriculaire (CIA), tétralogie de Fallot (Tdf), sténose pulmonaire, coarctation de l´aorte, transposition des gros vaisseaux (TGV) et sténose aortique (5%) [2]. Dans un quart des cas, la cardiopathie est associée à une ou plusieurs autres malformations congénitales [2]. La prise en charge des enfants souffrant de malformation cardiaque doit se faire tôt malgré les risques opératoires très élevés. L´importance des lésions résiduelles est fonction du type de cardiopathie mais aussi de l´âge auquel a eu lieu la correction chirurgicale: plus l´enfant est opéré tôt (< 3 ans), moins les séquelles sont importantes. Pour cette raison, on procède autant que possible à une correction totale dans la petite enfance et cette tendance offre aux enfants une qualité de vie quasi-normale [3]. Cependant la prise en charge de telles pathologies impose à l´anesthésiste une triple contrainte: pratiquer une anesthésie chez un enfant voir un nouveau-né, qui tous deux présentent des particularités anatomiques physiologiques et pharmacologiques différents de l´adulte. Maintenir en per opératoire une délicate balance entre les modifications hémodynamiques générées par la pathologie cardiaque et les mécanismes de compensation. Gérer en post opératoire des complications générées par la circulation extracorporelle. L´anesthésie pour chirurgie cardiaque pédiatrique a fait de tels progrès au cours de ces 25 dernières années permettant une réduction importante de la mortalité péri- opératoire. L´objectif de ce travail était d´évaluer la prise en charge anesthésique des cardiopathies congénitales opérées sous circulation extra corporelle (CEC) dans notre service après une première année d´activité et de comparer les résultats obtenus aux données de la littérature.

The article "Anaesthesia in on-pump cardiac surgery for congenital heart diseases at the Cuomo Pediatric Cardiology Center (Senegal)" was retracted in 2021. Reason: duplicate publication.

## Méthodes

Nous avons mené une étude rétrospective, descriptive sur une année allant de janvier à décembre 2017, dans le service de chirurgie cardiaque pédiatrique CUOMO de Dakar. Ont été inclus dans cette étude tous les patients opérés au cours de cette période pour une cardiopathie congénitale avec réalisation d´une circulation extracorporelle. Les patients opérés de pathologies rhumatismales ont été exclus de l´étude ainsi que les cardiopathies congénitales non opérées sous CEC.

Tous les patients inclus dans l´étude avaient bénéficié d´une consultation de cardiologie avec systématiquement un électrocardiogramme (ECG) et une échographie trans-thoracique. Ils bénéficiaient également d´une consultation de chirurgie cardiaque avant d´être envoyé pour la visite pré-anesthésique. Après confirmation de l´aptitude à l´anesthésie les patients étaient inclus au programme opératoire. Nous avons considéré comme facteurs de risque pour l´intervention chirurgicale les éléments suivants : une lésion cardiaque complexe, une malformation extra- cardiaque associée, une hypoxémie sévère (SpO2 < 80%), une viscosité sanguine trop importante (ht > 60%), une hypertension artérielle pulmonaire (HTAP) avec des résistances artérielles pulmonaires élevées (Rap/Ras > 0.5), une insuffisance ventriculaire, le jeune âge (< 3kg ou < 2 mois), une ischémie coronarienne.

Dès leur arrivée en salle d´opération les patients bénéficiaient systématiquement d´un monitorage à l´aide d´un électrocardioscope, une mesure de la pression artérielle non invasive et de la saturation périphérique en oxygène. Outre ce monitorage standard, les patients bénéficiaient systématiquement de la mise en place d´une voie veineuse centrale et d´un cathéter artériel. Ils servaient respectivement à la mesure de la pression veineuse centrale et de la pression artérielle invasive. Une échographie trans-œsophagienne était systématiquement réalisée en per opératoire soit par un cardiologue soit par le médecin anesthésiste.

En per opératoire une stratégie d´épargne sanguine était systématiquement réalisée par l´administration d´acide tranexamique. Une antibioprophylaxie était également réalisée. En fin d´intervention tous les malades étaient transférés systématiquement en réanimation intubés pour la suite de la prise en charge. Ils y bénéficiaient en post opératoire immédiat d´une échographie trans- thoracique.

The article "Anaesthesia in on-pump cardiac surgery for congenital heart diseases at the Cuomo Pediatric Cardiology Center (Senegal)" was retracted in 2021. Reason: duplicate publication.

## Résultats

Durant la période d´étude nous avons colligé 80 dossiers de patients opérés pour une cardiopathie congénitale. Pendant cette même période 136 patients avaient été opérés dans le service. La chirurgie des cardiopathies congénitales représente donc 58,8 % de l´activité chirurgicale. Parmi ces 80 patients, 60 ont été opéré sous CEC soit un taux de 75%. Pour les 20 autres patients souffrant de cardiopathies congénitales 17 ont bénéficié d´une cure de PCA et 03 d´une chirurgie palliative (02 interventions de Blalock et 01 cerclage de l´artère pulmonaire). L´âge moyen de nos patients était de 7,41 ans avec des extrêmes de 1 et 17 ans. Le poids moyen était de 21 kg +/- 10,8 kg avec des extrêmes de 7 et 60kg. Nous avons dénombré 27 patientes de sexe féminin et 33 de sexe masculin soit un sex-ratio de 1,22. Une notion de consanguinité avait été retrouvée chez 10 de nos patients soit une fréquence de 16,66% (Tableau 1). Nous avons recensé 22 cas de cardiopathies cyanogènes (36,66%) et 38 cas de cardiopathies non cyanogènes (63,34%) (Tableau 2). La cardiopathie non cyanogène la plus fréquente était la CIV (10 cas) et la cardiopathie cyanogène la plus fréquente était la tétralogie de Fallot (19 cas).

**Tableau 1:** répartition selon la consanguinité

Notion de consanguinité	nombre	pourcentage
oui	10	16,66%
non	50	83,34%
total	60	100%

**Tableau 2:** répartition des cardiopathies

Cardiopathies non cyanogènes	Cardiopathies cyanogènes
CIV 10 cas	Tétralogie de Fallot 19 cas
CIV + CIA 3 cas	CIA + retour veineux supra cardiaque 1 cas
CIV + sténose pulmonaire 1 cas	CIV + sténose pulmonaire 1 cas
CIV + membrane sous aortique 2 cas	Sténose pulmonaire 1 cas
CIV + sténose médioventriculaire 1 cas	
CIA 10 cas	
CIA + sténose pulmonaire 1 cas	
CAV 4 cas	
Sténose pulmonaire 1 cas	
Sténose médioventriculaire 1 cas	
PCA + membrane sous aortique 1 cas	
Membrane sous aortique 3 cas	

A l´examen clinique pré-opératoire aucune autre malformation n´était associée à la cardiopathie. Il n´était également pas retrouvé de critère prédictif d´intubation difficile chez nos patients. La saturation périphérique en oxygène dans les cardiopathies cyanogènes était en moyenne à 81% avec des extrêmes de 61% et 95%. Deux cas d´infections pulmonaires en cours avaient été notés lors de cet examen. L´ECG avait été réalisé chez tous les patients. Il était anormal dans 46 cas. Les anomalies retrouvées étaient: trouble du rythme (1 cas; arythmie complète par fibrillation atriale); trouble de la conduction (3 cas) hypertrophie de cavité (37 cas) trouble de la conduction associé à une hypertrophie de cavité (5 cas). Le bilan biologique retrouvait une anémie chez 2 patients en préopératoire. Neuf (09) patients présentaient un taux d´hématocrite élevé et 02 patients un trouble de l´hémostase associé à un hématocrite élevé. Il s´agissait dans tous les cas de patients souffrants de cardiopathie cyanogène. Aucun de nos patients ne présentait d´altération de la fonction rénale en préopératoire.

The article "Anaesthesia in on-pump cardiac surgery for congenital heart diseases at the Cuomo Pediatric Cardiology Center (Senegal)" was retracted in 2021. Reason: duplicate publication.

Un facteur de risque pour l´intervention avait été retrouvé chez 13 patients soit une fréquence de 21,7%. Parmi ces 13 patients, 12 souffraient d´une cardiopathie cyanogène (92,3%) et 1 d´une cardiopathie non cyanogène (7,7%). L´existence de certains de ces facteurs de risque ou d´une infection pulmonaire nécessitait une préparation des patients pour l´intervention. Ainsi 2 patients avaient bénéficié d´un traitement d´une hypertension artérielle pulmonaire (à base de sildénafil) et 2 autres d´un traitement pour une infection pulmonaire (antibiothérapie probabiliste). Au bloc opératoire l´induction anesthésique réalisée était inhalatoire dans 61,3% des cas et intraveineuse dans 38,7% des cas. Pour l´induction inhalatoire le sévoflurane était l´halogéné utilisé dans 100% des cas. Par contre l´induction intraveineuse présentait une grande variabilité des produits utilisés seuls ou en association. Le type d´entretien anesthésique réalisé en per opératoire était également variable d´un patient à l´autre. Il était fait avec des associations variables de morphiniques en bolus ou perfusion continue (fentanyl, sufentanyl), de curares, d´hypnotiques (propofol, benzodiazépines, halogénés). L´antibiotique utilisé était la céfazoline dans 53 cas (88,33%) et le céfuroxime dans 7 cas (8,83%).

La mesure de l´*Activated Clotting Time* (ACT) était variable chez les 60 patients opérés sous CEC. Chez 23 patients (38.3%) il était fait une mesure avant l´injection d´héparine, une trois minutes après l´injection d´héparine et une dernière mesure après antagonisation par la protamine. Le reste des patients (37) avaient bénéficié d´une seule mesure après injection d´héparine. La valeur de l´ACT avant la canulation aortique était en moyenne de 494.83 secondes avec des extrêmes de 276 et 999 secondes. Le volume d´amorçage de l´oxygénateur et des circuits de la pompe de CEC était fait avec des cristalloïdes ou colloïdes dans 57% des cas. Dans 43% des cas il y était associé des concentrés de culot globulaire. Tous les patients ont bénéficié d´une cardioplégie froide au sang dont la composition était variable en fonction des équipes. La température pendant la CEC était en moyenne de 34°5 Celsius et était mesurée au niveau rectal. Les extrêmes étaient de 24 et 36 degré. Un seul patient était opéré en hypothermie profonde à 24 degré avec arrêt circulatoire pour correction d´un retour veineux pulmonaire anormal total.

The article "Anaesthesia in on-pump cardiac surgery for congenital heart diseases at the Cuomo Pediatric Cardiology Center (Senegal)" was retracted in 2021. Reason: duplicate publication.

La durée de la CEC était en moyenne de 82,82 minutes +/- 33,41. Les extrêmes étaient de 30 minutes et 197 minutes. La durée moyenne du clampage aortique était de 58,31 minutes +/- 24,3. Les extrêmes étaient de 15 et 125 minutes. Nous avons noté la survenue d´une complication au cours de la CEC chez 4 patients soit une fréquence de 6,7%. Il s´agissait d´une hypotension persistante chez un patient et de 3 cas de fibrillation ventriculaire au moment de la reprise de l´activité cardiaque, nécessitant un choc électrique interne.

Des amines ont été utilisés chez 42 patients soit 70% de la population d´étude (60 patients). 34 patients ont bénéficié d´une association d´inotrope positif et vasoconstricteur; 6 patients uniquement des vasoconstricteurs; 2 patients uniquement des inotropes. En fin de CEC et après stabilisation de l´hémodynamique les patients étaient transférés en réanimation toujours intubés et sédatés. Il y était fait une échographie trans-thoracique de contrôle ainsi que des bilans biologiques. Lorsque leur état semblait stable l´extubation était alors envisagé. Le délai moyen pour l´extubation était de 12 heures avec des extrêmes de 6 heures et 7 jours. En post opératoire immédiat, une complication a été retrouvée chez 36 patients (60%). Il s´agissait de: Défaillance cardiaque gauche: 3 cas (8,33%); Défaillance cardiaque droite: 25 cas (69,44%); Hypertension artérielle pulmonaire: 4 cas (11.11%); Troubles du rythme: 1 cas (2,77%); Troubles de l´hémostase: 19 cas (52,77%), dont une thrombopénie dans 5 cas un taux de prothrombine bas dans 9 cas et une association des deux dans 5 cas (Le total dépasse 36 car les mêmes complications peuvent être retrouvées chez un même patient).

La durée moyenne d´utilisation des amines en réanimation était de 3 jours avec des extrêmes de 2 et 5 jours. L´évolution à court et moyen terme a été émaillée de complications en réanimation chez 3 patients (5%). Le premier patient avait été opéré pour une sténose pulmonaire; A j2 post opératoire il a présenté une défaillance cardiaque droite sévère avec un gradient ventricule droit- artère pulmonaire à 147mmhg. Il a été réintubé et a bénéficié d´un traitement à base de milrinone. Devant l´amélioration de la symptomatologie il a été extubé à j5 et transféré en hospitalisation à j13.

Le second patient avait été opéré pour un canal atrio-ventriculaire (CAV). L´évolution en réanimation a été marquée dans les premières heures par une hypoxie sévère. L´échographie réalisée au lit du malade a montré que la veine cave inférieure se drainait dans l´oreillette gauche responsable de l´hypoxie. La reprise chirurgicale a été faite à H3. L´évolution a été favorable et le patient a été transféré à j4 en hospitalisation. Le dernier patient avait été opéré pour une tétralogie de Fallot. Elle a présenté dans les heures suivant l´intervention un saignement important entrainant état de choc puis un arrêt cardiaque et son décès à H7. La mortalité au cours de la chirurgie des cardiopathies congénitales sous CEC était donc de 1,60%. La durée moyenne de séjour en réanimation était de 4,33 jours avec des extrêmes de 7 heures à 9 jours.

The article "Anaesthesia in on-pump cardiac surgery for congenital heart diseases at the Cuomo Pediatric Cardiology Center (Senegal)" was retracted in 2021. Reason: duplicate publication.

## Discussion

Dans notre étude nous avons colligé 80 dossiers de patients opérés pour cardiopathie congénitale sur une période d´une année. Seulement 60 d´entre eux ont été opérés sous CEC. Le nombre de patients opérés durant cette période était de 136. Dans une étude s´intéressant à la chirurgie des cardiopathies congénitales chez les adultes Haddad *et al*. [4] en 2015 avait retrouvé un total de 540 patients sur une période de 16 ans. Ce qui fait une fréquence d´environ 33 patients par année. Cette différence peut s´expliquer par le fait que la chirurgie des cardiopathies congénitales est plus fréquente et plus indiquée dans l´enfance. Aussi très peu de patients non opérés dans l´enfance atteignent l´âge adulte ou présentent des formes assez évoluées devenues alors inopérable. Seule une partie peut tirer encore profit de la chirurgie à cet âge. En 2011 Fall *et al*. dans une étude rétrospective s´intéressant à la prise en charge anesthésique et la réanimation des cardiopathies congénitales opérées par une équipe suisse à Dakar avait retrouvé 19 patients sur une période de 6mois [5].

L´âge moyen des patients opérés dans notre service était de 7,41 ans avec des extrêmes de 1 et 17 ans. Ces données sont toujours supérieures à celles recommandées dans la littérature (chirurgie avant 3 ans); ce qui limiterait le risque de séquelles et améliorerait la qualité de vie [3]. La difficulté principale que nous rencontrons dans la poursuite de cet objectif est double; d´abord le diagnostic des cardiopathies dans notre contexte se fait le plus souvent à un âge déjà avancé, mais aussi la prise en charge tant sur le plan anesthésique ainsi que les impératifs de la CEC des enfants en bas âge (< 2 mois ou 3kg) constituent un obstacle majeur. Cependant nous notons une nette progression dans la prise en charge de ces pathologies à Dakar car Fall *et al*. en 2011 avait retrouvé un âge moyen de 9,6 ans avec des extrêmes de 6 et 17 ans [5]. Nous avons dénombré 52,5% de patients de sexe féminin et 47.5% de sexe masculin pour toutes les cardiopathies congénitales opérées (avec ou sans CEC) dans le service durant la période d´étude. Ces chiffres sont sensiblement égaux à ceux trouvés par une étude belge réalisée par Moons *et al*. en 2002 [6]. Ils retrouvaient 51% de filles et 49% de garçons. Mbaye *et al*. [7] dans une étude faite à Dakar sur les cardiopathies congénitales chez des adultes trouvaient aussi une prédominance féminine (64%).

The article "Anaesthesia in on-pump cardiac surgery for congenital heart diseases at the Cuomo Pediatric Cardiology Center (Senegal)" was retracted in 2021. Reason: duplicate publication.

Dans notre étude nous avons retrouvé une notion de consanguinité chez 16,66% des enfants atteints de cardiopathies congénitales. La consanguinité est une source reconnue de survenue de tare génétique. Ceci renforce l´hypothèse selon laquelle une des causes de survenue de cardiopathie congénitale est d´ordre génétique. Fall avait retrouvé une fréquence de la consanguinité d´environ 15,78% [5]. Ces résultats sont proches de ceux que nous avons retrouvés. Les cardiopathies congénitales les plus fréquentes dans notre étude étaient la tétralogie de Fallot 31,66%; la CIA 16,66% et la CIV 16,66%. Dans d´autres études [8, 9] des prévalences différentes étaient retrouvées. Il y était fait une classification des cardiopathies congénitales les plus fréquentes pour 100 cas diagnostiqués. Venait alors en tête la CIV 26%, la CIA 12% et la PCA 8%. La tétralogie de Fallot qui était la plus fréquente dans notre étude y avait un taux de prévalence de seulement 8%.

L´examen clinique réalisé en préopératoire n´avait pas retrouvé de malformation associée à la cardiopathie. Cependant dans la littérature il est décrit que dans un quart des cas, la cardiopathie est associée à une ou plusieurs autres malformations congénitales [10]. L´ECG était normal chez 14 patients (23,33%). L´anomalie la plus retrouvée était une hypertrophie de cavité isolée chez 37 patients soit une fréquence de 46,25% (hypertrophie auriculaire ou ventriculaire). On retrouvait également un trouble de la conduction isolé ou associé à une hypertrophie de cavité chez 8 patients (bloc de branche droit ou gauche ou bloc bifasciculaire). Un trouble du rythme a été retrouvé chez un seul patient (1,25%). Il s´agissait d´une arythmie complète par fibrillation atriale. Par contre dans l´étude de Mbaye *et al*. [11] l´anomalie la plus retrouvée était le trouble du rythme à une fréquence de 18%. Le bilan biologique présentait une perturbation chez 13 patients (21,66%). Il s´agissait d´une anémie modérée chez 2 patients (7,5%). Onze patients (13,75%) présentaient un taux d´hématocrite élevé supérieur à 60%. Ces patients étaient tous porteurs de cardiopathies cyanogène. Cette polycythémie est due à la stimulation de la sécrétion d´érythropoïétine par l´hypoxie chronique [12]. Elle augmente de manière importante la viscosité du sang et implique souvent la présence de troubles de coagulation associés [12]. Ainsi retrouvions-nous parmi ces 11 patients 2 cas de troubles de la crase sanguine associés à l´hématocrite élevé.

The article "Anaesthesia in on-pump cardiac surgery for congenital heart diseases at the Cuomo Pediatric Cardiology Center (Senegal)" was retracted in 2021. Reason: duplicate publication.

Par ailleurs, la recherche de troubles électrolytiques et notamment le potassium, est recommandée chez les enfants recevant un traitement digitalique, diurétique et par inhibiteur de l´enzyme de conversion [12]. Dans notre étude nous n´avions pas retrouvé de cas de trouble ionique ni de perturbation de la fonction rénale. Dans notre étude nous avons retrouvé l´existence d´au moins un facteur de risque chez 13 patients soit une fréquence de 21,7%. Parmi ces 13 patients, 12 souffraient d´une cardiopathie cyanogène (92,3%) et 1 d´une cardiopathie non cyanogène (CIV + HTAP) (7,7%). Ces chiffres traduisent la difficulté que constitue la prise en charge des cardiopathies cyanogènes par rapport aux non cyanogène. L´existence de certains de ces facteurs de risque ou d´une infection pulmonaire imposait une préparation des patients pour l´intervention. La présence d´une infection récente des voies aériennes peut non seulement entrainer une hyperréactivité bronchique, mais aussi une modification des résistances vasculaires pulmonaires qui peut alors être mal tolérée chez les enfants porteurs de cardiopathies congénitales [12]. Ainsi 2 patients avaient bénéficié avant l´intervention d´un traitement pour une infection pulmonaire par une antibiothérapie. Deux autres patients présentaient une HTAP et ont bénéficié d´un traitement à base de sildénafil permettant d´abaisser les pressions pulmonaires avant la chirurgie.

Vingt à trente pour cent des enfants porteurs d´une cardiopathie congénitale présentent une insuffisance cardiaque au cours de leur évolution clinique [12]. Dans notre étude nous n´avons pas retrouvé de cas de décompensation cardiaque en pré-opératoire. Cela s´explique par le fait que les malades avant même d´être programmés pour la chirurgie sont suivis par une équipe de cardiologie. Celle-ci se chargeait de l´ajustement thérapeutique avant de référer les patients une fois que leur état semblait stable. L´induction réalisée était inhalatoire dans 61,3% des cas et intraveineuse dans 38,7% des cas. Pour l´induction inhalatoire le sévoflurane était l´halogéné utilisé dans 100% des cas. Par contre l´induction intraveineuse présentait une grande variabilité des produits utilisés seuls ou en association. Ceci s´explique par le fait que les équipes d´anesthésie variaient beaucoup. L´induction et l´entretien étaient faits non seulement en fonction des habitudes de chaque équipe mais également en fonction de la pathologie et de l´état clinique du patient. En effet Il n´y a pas de recette simple applicable à tous les enfants en anesthésie pour cardiopathies congénitales; l´extrême variabilité des pathologies fait que plusieurs techniques sont possibles, basées sur l´utilisation d´un agent principal et d´agents d´appoint. Le choix est guidé par la pathologie cardiaque, l´âge, la durée de la CEC, le degré d´hypothermie et les prévisions postopératoires [13].

The article "Anaesthesia in on-pump cardiac surgery for congenital heart diseases at the Cuomo Pediatric Cardiology Center (Senegal)" was retracted in 2021. Reason: duplicate publication.

Dans notre étude les patients ayant bénéficié d´une chirurgie sous circulation extra corporelle (60 patients) ont tous bénéficié d´une administration d´acide tranexamique en peropératoire. La technique d´administration de l´acide tranexamique en bolus ou en continue variait également d´une équipe à l´autre. Junejo *et al*. dans une étude comparant le bolus et la perfusion continue d´acide tranexamique pour la réduction du saignement chez des enfants bénéficiant d´une chirurgie pour cardiopathie congénitale cyanogène étaient parvenus à la conclusion qu´il n´existait pas de différence statistiquement et cliniquement significatif entre les 2 techniques [14]. Les paramètres qu´ils avaient étudiés étaient la quantité du saignement post opératoire et le temps de fermeture de la thoracotomie. Tous les patients opérés avaient bénéficié d´une antibioprophylaxie à base de céfazoline dans 90% des cas et de céfuroxime dans 10% des cas. La céfazoline est l´antibiotique recommandé dans la chirurgie cardiaque [15]. Le cefuroxime était utilisé faute de disponibilité de cefazoline. Nous avons noté un seul cas d´infection post opératoire (1,25%). Il s´agissait d´une sternite.

Nos patients bénéficiaient d´une injection de 300 UI/kg d´héparine et d´une mesure de l´ACT avant la canulation aortique. Le temps d´ACT recommandé est d´environ 400 secondes [16]. Dans notre étude le délai moyen de l´ACT était de 494.83 secondes. Ce qui correspond aux données de la littérature. Cependant certaines équipes procédaient à une mesure systématique de l´ACT avant l´injection d´héparine et d´une autre en fin de CEC après antagonisation par la protamine. Cette pratique permet de se rassurer sur la neutralisation de toute l´héparine administrée au patient mais également d´éliminé cette cause en cas de saignement post opératoire. Cependant elle reste limitée par la disponibilité des tubes à ACT.

Le volume de la CEC (amorçage ou priming) est 2 à 4 fois plus grand que le volume circulant de l´enfant. La dilution extrême imposée par le grand volume d´amorçage diminue la pression oncotique et l´hématocrite, ce qui augmente l´œdème tissulaire et baisse les résistances artérielles périphériques. Elle diminue la concentration des plaquettes et des facteurs de coagulation [10]. Pour réduire cette hémodilution il était associé dans 43% des cas des concentrés de culot globulaire et/ou du plasma frais congelé dans le priming de nos patients. Cette adjonction était surtout faite chez les enfants de moins de 5 ans chez qui l´hémodilution est plus important Tous nos patients ont bénéficié d´une cardioplégie froide au sang. La mise en évidence d´une supériorité de la cardioplégie au sang par rapport à la cardioplégie aux cristalloïdes a longtemps été l´objet de controverses. Cependant la cardioplégie au sang s´est progressivement imposée de sorte qu´elle ne se discute plus surtout dans les situations à risque (HVG, diminution de la fonction ventriculaire). Toutefois les mécanismes du bénéfice de la cardioplégie sanguine sur les vecteurs cristalloïdes restent incomplètement élucidés. On remarquera cependant qu´hémodilution et hypothermie se conjuguent pour limiter la quantité d´oxygène apportée au myocarde. De plus le cœur consomme l´oxygène en temps réel et on ne peut donc espérer la création d´un environnement aérobie que pendant les quelques minutes contemporaines de la perfusion de cardioplégie. Il est donc vraisemblable que les effets protecteurs de la cardioplégie au sang reposent sur les effets rhéologiques du sang et des effets cardioprotecteurs de certains de ses constituants (protéines, systèmes tampons, antioxydants) [10].

The article "Anaesthesia in on-pump cardiac surgery for congenital heart diseases at the Cuomo Pediatric Cardiology Center (Senegal)" was retracted in 2021. Reason: duplicate publication.

La température était en moyenne de 34°5 Celsius et mesurée au niveau rectal. Les extrêmes étaient de 24 et 36 degré. Un seul patient était opéré en hypothermie profonde à 24 degré avec arrêt circulatoire pour correction d´un retour veineux pulmonaire anormal total (RVPAT). La baisse du métabolisme cellulaire par le froid offre un certain degré de protection des organes et permet de prolonger le temps d´ischémie d´une durée variable selon la température [10]. Dans l´étude de Fall *et al*. la température moyenne en cours de CEC était de 35°C avec des extrêmes de 34 à 36°C [5]. Dans notre étude la durée de la CEC était en moyenne de 82,82 minutes + /- 33,41. Les extrêmes étaient de 30 minutes et 197 minutes. La durée moyenne du clampage aortique était de 58,31 minutes +/- 24,3. Les extrêmes étaient de 15 et 125 minutes. Il n´y a pas de durée maximale de CEC mais il est reconnu que la fréquence des complications augmente avec le temps [16]. Fall avait retrouvé des valeurs semblables avec un temps moyen de clampage aortique de 50mn et une durée moyenne de CEC de 90mn [5].

Au cours de la CEC les complications rencontrées dans notre étude sont: un cas d´hypotension persistante ayant nécessité des injections de vasoconstricteurs et trois cas de fibrillation ventriculaire lors de la reprise de l´activité cardiaque nécessitant des chocs cardiaques internes. Au cours de la chirurgie cardiaque l´utilisation des vasopresseurs et des agents inotropes pour la mise en charge est dictée par l´observation du cœur dans le champ opératoire et à l´ETO, par l´analyse des pressions artérielles et veineuses centrales, et par les modifications hémodynamiques imposées en fin de CEC [10]. Dans notre étude des amines ont été utilisés chez 42 patients soit 70% des patients: 34 patients ont bénéficié d´une association d´inotrope positif et vasoconstricteur; 6 patients uniquement des vasoconstricteurs; 2 patients uniquement des inotropes. Dans l´étude de Fall ML *et al*. 53% des patients avaient bénéficié d´amines [5].

The article "Anaesthesia in on-pump cardiac surgery for congenital heart diseases at the Cuomo Pediatric Cardiology Center (Senegal)" was retracted in 2021. Reason: duplicate publication.

En fin de CEC et après stabilisation de l´hémodynamique les patients étaient transférés en réanimation toujours intubés et sédatés. Il y était fait une échographie trans-thoracique de contrôle ainsi que des bilans biologiques. Lorsque leur état semblait stable l´extubation était alors envisagé. Le délai moyen pour l´extubation était de 12 heures avec des extrêmes de 6 heures et 7 jours. Selon certains auteurs une extubation rapide (< 4 heures post- opératoire) évite les complications liées à la ventilation mécanique (barotraumatisme, infections respiratoires, obstruction du tube endotrachéal); elle autorise une mobilisation précoce et raccourcit la durée de séjour en soins intensifs [10].

Bien que plaisante, cette théorie expose le patient à un risque d´hypoventilation ou un arrêt respiratoire. En somme, la durée de la ventilation mécanique postopératoire et le délai pour l´extubation font toujours débat, l´extubation sur table ou aux soins intensifs quelques heures plus tard ayant chacune leurs adeptes [17, 18]. Les complications les plus fréquentes en post CEC immédiat dans notre étude étaient la défaillance cardiaque droite (69,44%) les troubles de l´hémostase (52,77%) et l´HTAP (11,11%). Ces observations sont concordantes aux données de la littérature qui définissent la dysfonction droite comme étant la complication dominante [10].

L´évolution à court et moyen terme a été émaillée de complications en réanimation chez 3 patients (5%). Parmi ces 3 patients, 2 ont eu une évolution favorable. Le dernier patient est décédé, soit une mortalité de 1,6%. Haddad *et al*. [4] dans leur étude sur les cardiopathies congénitales à l´âge adulte retrouvaient une mortalité légèrement supérieure à 2,4%. Diouf [19] (1994) et Beye [20] (2010) dans des études réalisées également à Dakar chez des patients opérés pour des cardiopathies congénitales par des équipes étrangères retrouvaient respectivement des mortalités de 19% et 14%. Nos résultats témoignent des progrès réalisés dans la prise en charge des cardiopathies congénitales d´autant plus que les patients ont été opérés en majeure partie par l´équipe locale. La durée moyenne de séjour en réanimation était de 4,33 jours avec des extrêmes de 7 heures à 9 jours. Fall retrouvait une durée moyenne de séjour en réanimation de 6 jours [5]. Ceci témoigne d´une nette amélioration de la gestion post-opératoire de ce type de patients.

The article "Anaesthesia in on-pump cardiac surgery for congenital heart diseases at the Cuomo Pediatric Cardiology Center (Senegal)" was retracted in 2021. Reason: duplicate publication.

## Conclusion

Les cardiopathies congénitales sont complexes et très variables dans leur physiopathologie. Avec l´amélioration des techniques et des connaissances, leur morbi-mortalité a fortement diminué. Pour améliorer la prise en charge des enfants souffrants de ces pathologies une concertation entre l´anesthésiste le cardiologue pédiatre et le chirurgien est indispensable. Le choix d´une technique anesthésique pour un enfant porteur d´une cardiopathie sera fondé sur une bonne connaissance de la malformation et de ses répercussions, des effets cardiovasculaires et pulmonaires et des interactions éventuelles des agents à notre disposition. Un bon suivi en réanimation dans le post opératoire demeure capital pour une bonne évolution. Le diagnostic anténatal des malformations cardiaques permettrait d´améliorer cette prise en charge mais il reste encore aujourd´hui insuffisant dans nos contrées.

### Etat des connaissances sur le sujet

- Les cardiopathies congénitales sont des pathologies assez fréquentes dans nos contrées;
- Leur prise en charge chirurgicale est restreinte du fait du manque d´infrastructures adaptées, de personnel spécialisé dans ce domaine tant sur le plan anesthésique que chirurgical et cardiologique.

### Contribution de notre étude à la connaissance

- Elle nous permet de démontrer la faisabilité de la chirurgie cardiaque en Afrique avec des résultats similaire à ceux obtenus dans les pays développés;
- Elle démontre également que l´extrême variabilité des cardiopathies congénitales fait qu´il n´y a pas de recette d´anesthésie applicable à tous; le choix des produits anesthésiques et des catécholamines est guidé par la pathologie cardiaque, l´âge, la durée de la CEC, le degré d´hypothermie et l´hémodynamique postopératoire;
- La principale complication demeure la défaillance cardiaque droite (plus de 50% des cas) en fin de CEC.
